RETRACTED

# Bacteria-Induced Dscam Isoforms of the Crustacean, *Pacifastacus leniusculus*

**DOI:** 10.1371/journal.ppat.1002062

**Published:** 2011-06-09

**Authors:** Apiruck Watthanasurorot, Pikul Jiravanichpaisal, Haipeng Liu, Irene Söderhäll, Kenneth Söderhäll

**Affiliations:** 1 Department of Comparative Physiology, Uppsala University, Uppsala, Sweden; 2 National Center for Genetic Engineering and Biotechnology, National Science and Technology Development Agency, Pathumthani, Thailand; 3 State Key Laboratory of Marine Environmental Science, College of Oceanography and Environmental Science, Xiamen University, Xiamen, Fujian, People's Republic of China; Stanford University, United States of America

## Abstract

The Down syndrome cell adhesion molecule, also known as Dscam, is a member of the immunoglobulin super family. Dscam plays an essential function in neuronal wiring and appears to be involved in innate immune reactions in insects. The deduced amino acid sequence of Dscam in the crustacean *Pacifastacus leniusculus* (*Pl*Dscam), encodes 9(Ig)-4(FNIII)-(Ig)-2(FNIII)-TM and it has variable regions in the N-terminal half of Ig2 and Ig3 and the complete Ig7 and in the transmembrane domain. The cytoplasmic tail can generate multiple isoforms. *Pl*Dscam can generate more than 22,000 different unique isoforms. Bacteria and LPS injection enhanced the expression of PlDscam, but no response in expression occurred after a white spot syndrome virus (WSSV) infection or injection with peptidoglycans. Furthermore, *Pl*Dscam silencing did not have any effect on the replication of the WSSV. Bacterial specific isoforms of *Pl*Dscam were shown to have a specific binding property to each tested bacteria, *E. coli* or *S. aureus*. The bacteria specific isoforms of *Pl*Dscam were shown to be associated with bacterial clearance and phagocytosis in crayfish.

## Author Summary

Invertebrate animals lack an adaptive immune system and have no antibodies. Vertebrate antibodies belong to the immunoglobulin super family of proteins, and one other member of this large family is the Down syndrome cell adhesion molecule or *Dscam*. Of specific interest is that Dscam proteins in invertebrates show a great diversity of isoforms, and its gene structure in *Drosophila melanogaster* and other insect species allow for more than 30,000 different isoforms. Dscam proteins are important for the interaction between neurons in insects, but recently a role for this hypervariable protein in immune defense has been shown. Here, we show that Dscam proteins with similar highly variable structures are present in a crustacean, the freshwater crayfish *Pacifastacus leniusculus*. We also found that specific isoforms could be induced in the animal after injection of different bacteria. The Dscam isoforms induced by *Escherichia coli* were found to cluster together in a phylogenetic analysis. Furthermore we produced recombinant proteins of the different isoforms that were induced by *E. coli* and *Staphylococcus aureus* and we could demonstrate that these proteins can bind specifically to their corresponding bacteria. The bacteria specific isoforms of Dscam were also shown to be associated with bacterial clearance and phagocytosis in crayfish. Our study therefore provides new insights into the function of invertebrate Dscams in immunity.

RETRACTED

## Introduction

The immunoglobulin super family (IgSF) is composed of proteins that contain at least one immunoglobulin domain [1]. Several members of IgSF are expressed on the cell surface and there serve as receptors for diverse ligands, and contribute to a variety of cellular activities [2]. In vertebrates, many IgSF members play essential roles as immune molecules (also known as antibodies) by recognizing non-self entities and then promoting their elimination [3]. Although it appears as if all invertebrates lack true antibodies, diversified IgSF molecules have been shown to be involved in immune defense of several invertebrates [4], [5]. However, this does not imply that the diversification of IgSF in invertebrates have any relation to the antibody diversification in vertebrates [5]. Recently, one IgSF member, the Down syndrome cell adhesion molecule gene or *Dscam*, that can generate hypervariable isoforms through alternative splicing was shown to act as an opsonin and to enhance phagocytosis in insects [4], [6].

*Dscam* was first detected on the human chromosome 21q22, a region associated with Down Syndrome [7]. Then, orthologues of Dscam were identified in various species and the typical domain structure of the *Dscam* gene is highly conserved. The Dscam molecules are widely expressed in the nervous system and play an essential role in neural circuit formation [8], [9]. Moreover, transcripts of fly Dscam was detected in fat body cells and hemocytes, which both are important components of the insect immune system [4], [10]. The Dscam in hemocytes of *Drosophila melanogaster* and *Anopheles gambiae* can bind to *Escherichia coli* and potentially acts as both a phagocytic receptor and as an opsonin. In the mosquito, *Dscam* can generate pathogen-specific spliced forms upon immune challenge [6]. These findings provide some evidences that Dscam may have functions not only in neuronal wiring, but also in innate immunity in insects.

In the present study, the full-length cDNA and variable regions of *P. leniusculus* Dscam (*Pl*Dscam) were identified and characterized. We also present results showing that different isoforms of *Pl*Dscam can be induced by immune challenge, that they can bind bacteria and that they are important in bacterial clearance.

RETRACTED

## Results

### Isolation and characterization of the *Pl*Dscam

A large open reading frame of *Pl*Dscam (6,009 bp) was identified that encodes a polypeptide of 2,002 aa (Figure 1A). The closest sequence matching that of *Pl*Dscam was Dscam of *L. vannamei* (identity * = *85%). Domain homology analysis using SMART showed that the deduced amino acid sequence contains a signal peptide at amino acids 1–24, ten tandem repeated immunoglobulin domains (Ig), six fibronectin type III domains (FNIII) and a transmembrane domain (TM). The domain organization of *Pl*Dscam is 9(Ig)-4(FNIII)-(Ig)-2(FNIII)-TM (Figure 1B). It also has a conserved cell attachment sequence (Arg-Gly-Asp: RGD motif) between Ig6 and Ig7 (Figure 1A). The sequence in the 3′ UTR contains a polyadenylation signal (AATAA) and is located at 55 bp upstream of the poly A tail (Figure 1C).

**Figure 1:** Identification and characterization of Dscam in *P. leniusculus*. A) Amino acid sequence of *Pl*Dscam; double underlining represents signal peptide, while the Immunoglobulin (Ig) and Fibronectin type III (FNIII) domains are indicated by light and dark gray shading, respectively. A conserved RGD motif between Ig6 and Ig7 is indicated by single underlining. In addition, the single transmembrane domain is shown in a box. B) Schematic diagram showing the domain organization of the *Pl*Dscam protein. C) 3′ UTR containing the polyadenylation signal (AATAA) is indicated by double underlining and a stop codon is bold and underlined.

### Expression of *Pl*Dscam transcript diversity

To identify the variable regions of *Pl*Dscam, several regions of the *Pl*Dscam were amplified using different primer pairs and the location of each pair of primers is shown in Figure S1. Fifty clones of each of the six amplified regions were selected and sequenced, translated and aligned using ClustalW. Alternatively spliced mRNA segments of the *Pl*Dscam were detected in the N-terminal of Ig2 and Ig3, in the entire length of the Ig7 domain, in the transmembrane domain and in the cytoplasmic tail (Figure 2B–E and Figure S1A). In total 12, 29, 32 and 2 alternative spliced forms of the exons encoding Ig2, Ig3, Ig7 and the transmembrane domains, respectively were detected and therefore at least 22,000 different unique isoforms could in theory be generated (Figure 2A–2E). The other domains were highly conserved, especially Ig8-FNIII4. The cytoplasmic tail of *Pl*Dscam contains some highly conserved motifs similar to the corresponding area in Dscams of other species (Figure S1B).

RETRACTED

**Figure 2:** High diversity regions of Dscam in freshwater crayfish. A) Diagram showing the locations of putative alternatively spliced exons of *Pl*Dscam. The variable regions are indicated at the N-terminal parts of Ig2 (red) and Ig3 (pink) and complete Ig7 (blue) and transmembrane (green) domains in crayfish. The number of alternative exons is presented by bars under the diagram. B–E) Multiple amino acid sequence alignment of *Pl*Dscam variable regions of Ig2(B), Ig3(C), Ig7(D) and transmembrane domain (E) aligned by ClustalW, Dark shading indicates the boundary of each domain.

### Tissue expression and phylogenetic analysis of *Pl*Dscam

In crayfish, *Pl*Dscam was abundantly expressed in the heart, moderately expressed in the testis, the hematopoietic tissue (HPT), brain and nerve, whereas low expression was detected in the stomach, gill, muscle and hemocytes. The *Pl*Dscam was not detected in hepatopancreas or in intestine (Figure 3A).

**Figure 3:** Tissue distribution and phylogenetic analysis. A) The expression of *Pl*Dscam was studied in various tissues, such as HP  =  Hepatopancreas, ST =  Stomach, IN =  Intestine, G =  Gill, TT =  Testis, H =  Heart, M =  Muscle, B =  Brain, HC =  Hemocyte and N =  abdominal nerve. A 40S ribosomal gene was used as an internal control. B) A phylogram based on multiple alignments between *PlDscam* and other Dscam proteins; *Drosophila melanogaster* (AAF71926), *Apis mellifera* (AAT96374), *Homo sapiens* (AF217525), *Mus musculus* (NP_112451), *Danio rerio* (AAT36313), *Daphnia pulex* (ACC65888), *Xenopus tropicalis* (NP_001136135), *Gallus gallus* (XP_416734), *Bos taurus* (XP_002693048), *Canis familiaris* (XP_546506) *Rattus norvegicus* (AAL57167), *Macaca mulatta* (XP_002803170), *Callithrix jacchus* (XP_002761477), *Tribolium castaneum* (NP_001107841), *Nasonia vitripennis* (XP_001599258), *Acyrthosiphon pisum* (XP_001949262), *Equus caballus* (XP_001491675), *Aedes aegypti* (EAT37388), *Aplysia californica* (ABS30432) and *Litopenaeus vannamei* (ACZ26466). A human junctional adhesion molecule A or JAMA was used as outgroup (NP_058642).

A phylogenetic analysis clearly separated the Dscam proteins of vertebrates and invertebrates in two different groups and *Pl*Dscam clustered with other members of invertebrate Dscams (Figure 3B).

### LPS and bacteria injection induce *Pl*Dscam transcription

To investigate whether immune challenge induces higher expression of *Pl*Dscam in crayfish hemocytes, LPS, peptidoglycan (PG), *E. coli*, *S. aureus* or WSSV was used as immune elicitors. The results of quantitative RT-PCR revealed that the *Pl*Dscam mRNA expression was significantly induced by LPS-, *E. coli-* and *S. aureus* at 6 h to 24 h post injection compared to controls (Figure 4A, 4C, 4D). In contrast, the expression profile of *Pl*Dscam in PG- and WSSV- injected animals was not changed (Figure 4B and 4E).

RETRACTED

**Figure 4:** Expression profiles of *Pl*Dscam in response to immune challenge. *Pl*Dscam expression was significantly higher than the control from 6 h post-injection with LPS (A), *E. coli* (C) and *S. aureus* (D). In contrast, PG (B) and WSSV (E)-injection did not have any effect on the *Pl*Dscam expression level. The asterisk indicates that the expression levels are significantly different (*P<0.05, **P<0.01).

### Clustering of *Pl*Dscam isoforms in hemocytes during a bacterial infection

In order to characterize the major isoforms of *PlDscam* in hemocytes of normal and bacteria injected crayfish, *Pl*Dscam cDNA fragments encompassing the signal peptide to Ig3 from each group were amplified and cloned (Figure 5A). A total of 50 clones of each cDNA fragment were sequenced. Ten isoforms were detected in all groups, i.e. normal, *E. coli* injected and *S. aureus* injected crayfish. These isoforms were named as Normal isoform (N) (Table S2 and Table S3). Furthermore ten abundant isoforms were found only in the *E. coli* or *S. aureus* injected group and were named *E. coli* induced isoform (E) or *S. aureus* induced isoform (S), respectively (Table S2 and Table S3). All isoforms were subjected to multiple sequence alignment using clustalW. The similarity of each *Pl*Dscam isoform was then clustered by the maximum likelihood (ML) and Bayesian inference (BI) methods. As shown in Figure 5B, the clustering tree contained two major branches. The *E. coli* induced isoforms were separated into one branch, whereas the other branch consisted of two sub-branches of normal isoform and *S. aureus* induced isoform (Figure 5B).

**Figure 5:** Bacteria-induced *Pl*Dscam isoforms. A) Different isoforms of *Pl*Dscam were amplified from hemocyte cDNA of normal crayfish, at 12 h post injection with *E. coli* or *S. aureus*. The PCR products were detected on 1.2% agarose gel. The PCR-products from normal crayfish (N) are shown in lanes 1–3, while PCR-products from *E. coli* (E) and *S. aureus* (S) injected animals are shown in lanes 4–6 and 7–9 respectively. B) Clustering of all *Pl*Dscam isoforms is based on the similarity of their amino acid sequence. The gray shaded boxes represent the chosen isoforms. C) Multiple amino acid sequence alignment of the isoforms E2, N6 and S9 aligned by ClustalW. Dark shading indicates the boundary of each domain.

The E isoforms of PlDscam isoforms had a VNKEYIIRGDSA(F/I)LKCSIPSFVA(D/N) motif and a EIGSPATFTCRAQAHPVPQY motif present at the N-terminal of the Ig2 and Ig3 domains, respectively. As shown in Figure 5B and 5C the isoforms N6, E2 and S9 are different, and therefore we used these isoforms as representative alternative spliced forms of normal, *E. coli*- and *S. aureus*-induced isoforms for a bacterial binding assay.

RETRACTED

### Binding of r*Pl*Dscam to *E. coli* and *S. aureus*

Recombinant proteins covering the Ig1-Ig3 domains of the *P*lDscam isoforms of N6, E2 and S9 were produced and tested whether these domains have any putative function in binding to *E. coli or S. aureus*. These proteins were expressed in bacterial systems and the size of all soluble recombinant proteins was ∼67 kDa (Figure 6A). All recombinant proteins were fused with GST at the N-terminus and contained the Ig1-Ig3 domains. We used these r*Pl*Dscams in bacterial binding assays to reveal whether different isoforms are capable of direct binding to bacteria. The GST protein was used as a non-specific binding control in these experiments. The *in vitro* bacterial binding assays showed that all isoforms of *Pl*Dscam had different binding ability to the two tested bacteria. The r*Pl*Dscam of isoform E2 clearly bound to *E. coli* and had significantly higher binding than the N6 and S9 isoforms. In contrast, binding of r*Pl*Dscam S9 to *S. aureus* was significantly higher (P<0.05) than that of N6 and E2 (Figure 6B).

**Figure 6:** Bacteria-induced *Pl*Dscam isoforms have different binding ability to bacteria. A) Different *Pl*Dscam isoforms were amplified from N6, E2 and S9 subclones and recombinant proteins were produced. The recombinant isoforms were subjected to 12% SDS and were confirmed by western blotting. Isoforms from non-injected animals in lanes 1 and 4; *E. coli*- induced isoform in lanes 2 and 5; and *S. aureus*-induced isoform in lanes 3 and 6. B) *In vitro* binding assays of r*Pl*Dscam isoforms of *E. coli* (left) and *S. aureus* (right), respectively. Binding of bacteria to different r*Pl*Dscam isoforms, consisting of N6 = isoforms from non-induced animal, E2 =  *E. coli* induced isoforms, S9 =  *S. aureus* induced isoforms or GST =  control recombinant protein was determined using ELISA by measuring the absorbance of samples at 450 nm (OD450). C and D) The effect of bacteria induced isoforms on the clearance process *in vivo* was tested by pre-incubation of the bacteria *E. coli* (C) and *S. aureus* (D) with each recombinant isoform prior to injection into crayfish. The bacterial numbers in crayfish were determined as CFU/ml of crayfish in the hemolymph at 40 min (black) and 3 h (grey) after the bacterial challenge. This experiment was repeated three times and data represent means of these experiments. E) Phagocytosis and nodule formation of FITC-conjugated heat-killed bacteria by crayfish hemocytes. Black arrows show nodule formation under normal light microscopy. White arrows show the ingested FITC-conjugated heat-killed bacteria by crayfish hemocytes under UV light microscope. Red arrows show nodules that contain several ingested bacterial particles under UV light microscope. F) The percentage of crayfish hemocytes ingesting FITC-conjugated heat-killed *E. coli* (left) and *S. aureus* (right) that had been pre-incubated with each isoform of the recombinant proteins and the phagocytic hemocytes was determined at 1.5 h after challenge. Significant difference compared to control is marked by * = P<0.05 and **  = *P<0.01*.

RETRACTED

### The effect of specific bacteria induced isoforms on bacterial clearance and phagocytosis

Recombinant proteins of isoforms E2 and S9 that specifically interacted with *E. coli* and *S. aureus*, respectively, were found to interfere with bacterial clearance and phagocytosis in crayfish. Pre-incubation of *E. coli* with E2 followed by injection into the animals did increase the number of bacteria in circulation (Figure 6C). Similarly with *S. aureus*, the number of bacteria was the highest in the S9 isoform of r*Pl*Dscam pre-incubated group (Figure 6D). This result clearly indicates that the specific r*Pl*Dscam could interfere with bacterial binding to the hemocytes. These results were in agreement with the phagocytosis assay, since if *E. coli* and *S. aureus* were coated with the E2 and S9 isoforms respectively, this resulted in a significant decrease in the phagocytic activity (Figure 6F).

### *In vitro* effect of *Pl*Dscam gene silencing on WSSV replication

The role of *Pl*Dscam during a WSSV infection was investigated using *Pl*Dscam RNAi to suppress the *Pl*Dscam expression. The *Pl*Dscam gene was completely knocked down in an HPTcell culture (Figure 7A) whereas the 40S ribosomal gene was unaffected. However, *Pl*Dscam silencing did not have any effect on WSSV replication as shown with no changes in transcription level of WSSV structural protein transcript VP28 between control and *Pl*Dscam silenced groups (Figure 7B and 7C). Moreover, this result also indicates that the expression of *Pl*Dscam was not affected by WSSV infection. This agrees with our previous experiment where we injected WSSV to live crayfish and the transcript level of Dscams was not affected (Figure 4E).

**Figure 7:** Effect of *Pl*Dscam silencing on viral replication of WSSV *in vitro*. A) Silencing of *Pl*Dscam using dsRNA in cultured HPT cells was confirmed by RT-PCR before WSSV inoculation. B) WSSV VP28 expression in *Pl*Dscam silenced animals (lane 7–9) and the control (lane 4–6). UV-killed WSSV was served as control (lane 1–3), analyzed by semi-quantitative RT-PCR. C) Statistical analysis after comparing different band intensity of the results shown in (B). Significant differences are indicated by asterisks (*P<0.05*).

RETRACTED

## Discussion

The typical domain structure of Dscam with an extracellular domain, a single transmembrane domain and a C-terminal cytoplasmic tail, is highly conserved within arthropods and vertebrates [7], [11]. This domain architecture was also found in *Pl*Dscam. Diversity in *Dscam* is generated through alternative splicing and variable alternative exons were found in the N-terminal half of Ig2 and Ig3, in the entire Ig7 domain and in the complete transmembrane domain [12]. These four variable domains are highly conserved within arthropods, including the *Pl*Dscam. It is noticeable that the alternative splicing of these exons clearly contributes to separate Dscam of vertebrates from invertebrates in our phylogenetic analysis [11].

The Dscam was initially identified for its essential roles in neuronal wiring, so its transcript is present in high quantity in neuronal organs [13]. The *Pl*Dscam was also detected in the neural system of crayfish. However, recently a putative role of Dscam in host defense was shown in *D. melanogaster* and *A. gambiae* [4], [6]. Both *D. melanogaster* and *A. gambiae* Dscams were required for host resistance and phagocytosis of bacteria [14]. Dscams of the mosquito respond to pathogen infection by generating specific isoforms and these pathogen-specific isoforms of Dscam can bind directly to pathogens [15]. The response of IgSF molecules to pathogens does not only generate specific isoforms, but also an increase in the number of these isoforms, such as is the case with the fibrinogen-related proteins (FREPs) in snails [5]. FREP production is enhanced following parasitic invasion, and these proteins can bind to parasitic invaders or their products. In crayfish challenge with both Gram-negative and Gram-positive bacteria induced higher transcription of *Pl*Dscam. A high transcription of *Pl*Dscam was obtained after LPS injection, whereas PG or viral injection of WSSV had no such effect. Most Gram-positive bacterial cell walls or cell membranes contain several components, including PG, lipoteichoic acid (LTA), and lipoproteins [16]. The high transcription of *Pl*Dscam achieved as a response to *S. aureus* injection but no response to PG may indicate that the *Pl*Dscam respond to other components of the *S. aureus* cell wall, such as LTA which has similar physiochemical properties to LPS from Gram-negative bacteria [17].

RETRACTED

Previous results from *D. melanogaster* and *L. vannamei* showed that the hemocytes of immune challenged animals exhibited higher variability of the Ig2 and Ig3 domains but only a few Ig7 variants compared to normal animal [4], [18]. This is the reason why we studied bacteria specific induced isoforms and produced recombinant proteins covering only the Ig1-Ig3 region. Interestingly, *Pl*Dscam isoforms of *E. coli* injected crayfish mainly encoded “VNKEYIIRGDSA(F/I)LKCSIPSFVA(D/N)” and “EIGSPATFTCRAQAHPVPQY” motifs at the N-terminal part of the Ig2 and Ig3 domains, respectively. This implies that these two motifs might be important parts of the specific *Pl*Dscam isoforms in *E. coli*-infected crayfish. This is consistent with results from our bacterial binding assay, which showed that the recombinant proteins containing these two motifs (E2), could bind to *E. coli* better than the other isoforms (N6 and S9). In addition, binding of *S. aureus*-induced isoforms (S9) to *S. aureus* was also higher than E2 and N6. These results indicate that the pathogen induced isoforms of *Pl*Dscam have a specific binding property to each type of challenged bacteria. This specific interaction may be associated with some immune defense reaction as shown with mosquito Dscam [6]. To address this question, recombinant proteins (N6, E2 and S9) were pre-incubated with bacteria or FITC conjugated heat killed bacteria to study bacteria clearance and phagocytosis *in vivo*. When, the bacteria-induced *Pl*Dscam isoforms were coated on *E. coli* or *S. aureus* and then injected into live animals, this resulted in lowered clearing rates of bacteria in the hemolymph. This implies that the specific *Pl*Dscam fragments covered the binding sites of the bacteria so they could not bind to the membrane bound *Pl*Dscam on the hemocytes and hence the bacterial number increases since the clearance of bacteria by phagocytes is inhibited.

In the case of mosquito, *Ag*Dscam is not only a determinant of resistance to bacteria but also affects the resistance towards the malaria parasite *Plasmodium* [6]. This implies that Dscam might be involved in other host pathogens reactions in crayfish. The Dscam belongs to a subfamily of the Immunoglobulin super family (IgSF). Indeed, many members of IgSF proteins have been reported to interact with and promote entry of numerous virus, including for example the junctional adhesion molecule A (JAM A), that could bind with and facilitate entry of reovirus [19], [20]. So, it is possible that *Pl*Dscam could bind to virus like the other members of IgSF and maybe facilitate entry of virus into crayfish hemocytes. WSSV is a virulent pathogen that causes death in many species of crustaceans such as crayfish [21] and therefore we tested a possible relationship between *Pl*Dscam and this important arthropod virus. We performed experiments to reveal whether WSSV challenge could increase transcription of *Pl*Dscam and whether *Pl*Dscam RNAi had any effect on WSSV replication. However, we could not detect any increase in *Pl*Dscam mRNA expression after WSSV infection, and more important, if the *Pl*Dscam gene was completely silenced this could not affect WSSV infection or replication.

RETRACTED

## Materials and Methods

### Crayfish

Healthy intermolt freshwater crayfish (*P. leniusculus*) were obtained from Lake Hjälmaren, Sweden and maintained in aerated tap water at 10°C.

### Cloning of full length *PlDscam* cDNA

Total RNA (at least 1 µg) was extracted from the heart and converted into cDNA using ThermoScript (Invitrogen). The degenerate primers were designed from the conserved region of insect Dscam including *Drosophila*, *Apis*, *Aedes* and *Tribolium* (DSCAM-e5 F: 5′-AARCAYMGIYTIACIGGIGARAC-3′; DSCAM-e7 R: 5′-GTI ARIACIGTYTCIACI SWYTC-3′). The resulting PCR product was purified and cloned into a TOPO vector (Invitrogen) and sequenced. A partial sequence was used for the further step. Gene specific primers for Rapid amplification of cDNA ends (RACE) technique (Table S1) were designed from the partial sequence and 5′ or 3′ RACE-PCR was performed with a SMART universal primer A mix (SMARTer RACE cDNA Amplification Kit user manual, Clontech). Thermal cycling was as follows: 25 cycles of 94°C 30 s, 68°C 30 s, and 72°C 3 min. The 5′ and 3′ RACE PCR products were cloned into TOP10 vector and sequenced.

### *Pl*Dscam sequence analysis and phylogenetic analysis

The nucleotide sequence of *Pl*Dscam was compared to others in Genbank using BlastX. Multiple sequence alignment was done by ClustalW (http://www.ebi.ac.uk/Tools/clustalw/index.html). The deduced amino acid domain was predicted with SMART (http://smart.embl-heidelberg.de/). A phylogenetic tree representing the relationship between *Pl*Dscam and other proteins was analyzed by the maximum likelihood (ML) and Bayesian inference (BI) methods. A PhyML program (under the Whelan and Goldman (WAG) and gamma model with four categories) was used in ML analysis [22]. For the BI method, we used MrBayes program [23] with CAT model (3,000 cycles, first 1,000 cycles removed as burn-in, and the analysis was repeated three times with identical results). Internal blanch support values was from analysis of 1,000 ML bootstrap replicates. This evolutionary phylogram was based on the conserved region of Dscam from Ig8 to FNIII4, whereas phylogram for clustering of all *Pl*Dscam isoforms was based on the similarity of their amino acid sequence and were used with the same methods as described above.

RETRACTED

### Tissue distribution of *Pl*Dscam mRNA

RNA from various tissues, including hepatopancreas, stomach, intestine, heart, hematopoietic tissue (Hpt), muscle, brain, hemocytes and nerves, was extracted following the instruction of GenElute Mammalian Total RNA Miniprep kit (Sigma) followed by treatment with RNase-Free DNase I (Ambion, Austin, TX). Complementary DNA was synthesized using ThermoScript. *Pl*Dscam gene specific primers (GSP-*Pl*Dscam-F, 5′- TGGGAAGTGATGCCAGGTTAGA-3′; GSP-*Pl*Dscam-R, 5′-TTGAATCAGCAGACATAACCAAAGC-3′) were designed from full-length cDNA of *Pl*Dscam and its PCR product covered the conserved Dscam region (from Ig8 to FNIII3). A 40S ribosomal gene was used as internal control in all PCR experiments and its specific primers (40S-F, 5′-CCAGGACCCCCAAACTTCTTAG-3′; 40S-R, 5′-GAAAACTGCCACAGCCGTTG-3′) were designed from *P. leniusculus* Lamda Zap Express library Hpt cDNA (Genbank accession no. CF542417). PCR conditions were as follows: 94°C 2 min, followed by 30 cycles of 94°C 20 s, 58°C 20 s, and 72°C 1 min for the *Pl*Dscam gene and 25 cycles for 40S ribosomal gene. The PCR products were analyzed on 1.2% agarose gel stained with ethidium bromide.

### Identification of alternatively expressed regions in *PlDscam*

Due to the large size of full length of *PlDscam*, it was necessary to use several pairs of primers for identification of the different variable regions. PCR of each region was performed with gene specific primers (Table S1) and thermal cycling was as follows: 94°C 2 min, followed by 30 cycles of 94°C 20 s, 60°C 20 s, and 72°C 1.30 min. The PCR products from four different tissues, such as heart, brain, hemocytes and HPT, were cloned into TOP10 vector and 25 individual clones from each tissue were sequenced.

### Immune challenge, sample collection and *Pl*Dscam transcription analysis

*E. coli* and *S. aureus* were cultured in LB broth at 37°C until OD _600_ was ca 0.5. The bacteria were washed three times with 0.85% NaCl by centrifugation at 900 g for 10 min at room temperature. The pellets were resuspended in sterile 0.85% NaCl and adjusted to an approximate concentration of 2×10^8^ CFU/ml. Two groups of three crayfish were injected in the base of the forth walking leg with 100 µl of *E. coli* and *S. aureus*, respectively (approximately 2×10^7^ CFU/crayfish). The control group was injected with 100 µl of 0.85% NaCl.

WSSV was purified with a method described by Xie et al.[24]. The purified virus was resuspended in sterile crayfish saline buffer (CFS: 0.2 M NaCl, 5.4 mM KCl, 10 µM CaCl_2_, and 10 mM MgCl_2_, 2 mM NaHCO_3_, pH 6.8) at a concentration of 2×10^7^ copies/ml. One hundred microliter of WSSV (equivalent to 2×10^6^ copies) or CFS (as control group) was injected as previously described. The experimental setup was made in triplicates.

RETRACTED

Two groups of three crayfish received injections with 100 µl lipopolysaccharides (LPS: Sigma, from *E. coli*) or peptidoglycan (PG: Sigma, from *S. aureus*) in a sterile CFS with a concentration of 0.2 mg/ml. One hundred microliter of CFS was used for the controls.

Hemolymph of crayfish from all experiments was collected at 0, 6, 12 and 24 h post injection and the hemocytes were separately isolated for RNA extraction. The transcript levels of *Pl*Dscam were detected by quantitative RT-PCR using the QuantiTect SYBR green PCR kit (QIAGEN). The expression of PlDscam was normalized to the expression of the mRNA encoding the crayfish ribosomal protein gene (R40s) for each sample. The primers used are shown in Table S1. The qPCR reactions contained 5 µl of 1∶10 diluted cDNA template, 1× QuantiTect SYBR Green PCR master mix (QIAGEN) and 5 µM forward and reverse primers in a 25-µl reaction volume. The following amplification profile was used: 95°C for 15 min, followed by 45 cycles of 94°C for 15 s, 58°C for 30 s, and 72°C for 30 s. All qPCR reactions were performed in duplicate. The hemocytes from a least three crayfish were used for each time point.

### Transcription analysis of *Pl*Dscam isoforms in response to *E. coli* and *S. aureus*

The variable region, from the signal peptide to the Ig3 domain region, was amplified from hemocyte cDNA templates from groups of crayfish injected with *E. coli* or *S. aureus*, respectively, and the control group at 12 h post injection with F1 and R2 primers (Table S1). The PCR products from each of these groups were subcloned into TOP10 vector and fifty colonies of each group were sampled and subsequently sequenced. Multiple sequence alignment was done by ClustalW and clustering tree of the different isoforms was constructed as described above.

### Recombinant protein of the *Pl*Dscam isoforms

The ORFs without the signal peptide encoding different *Pl*Dscam isoforms were amplified from the original templates N4, E1 and S7 with Dscam-expression-BamHI-Forward (5′-TTTTGGATCCAACCCGACAACCGTGTGGACTTCA-3′) and Dscam-expression-XhoI-Reverse (5′- TTTCTCGAGCCAGGTAACAGACTTGACGGGGTTG-3′) primers. The resulting insert was cloned into pGEX-4T-1(GE healthcare) at BamHI and XhoI and transformed into BL21 *E. coli*. Single colonies were grown in LB medium containing 100 µg/ml ampicillin to OD_600_ = 0.6 and induced with 1 µM IPTG for 5 h at 37°C. The protein was expressed as a fusion product with a glutathione S-transferase part at the N-terminus of r*Pl*Dscam. After purifying this GST-fusion protein on a GST-trap FF column (GE healthcare), the presence of the recombinant protein was confirmed by western blot. The protein samples were subjected to 12% SDS-PAGE and then transferred electrophoretically to PDVF membranes. The membrane was blocked by immersion in 10% skimmed milk in TBST for 1 h and washed three times in 1 x TBST (10 mM Tris-HCl, pH 7.5, containing 150 mM NaCl and 0.1% Tween 20). The membrane was then incubated with 1: 2,000 dilution of a primary antibody for GST (Sigma) in TBST for 1 h. Then, the previous washing procedure was repeated before the membrane was incubated with anti-mouse-IgG peroxidase-linked species-specific whole antibody from sheep (GE Healthcare) at 1: 3,000 in 1xTBST for 1 h and washed with TBST for 3×10 min. For detection, the ECL Western blotting reagent kit (Amersham Biosciences) was used according to the manufacturer's instructions.

RETRACTED

### Bacterial binding assay

A bacterial binding assay was modified from the method described by Yu et al.[25] Briefly, *E. coli* or *S. aureus* was prepared as previously described. An aliquot 100 µl of the bacteria was immobilized on 96 well plates at approximately 10^8^ CFU/well by incubating for 30 min at room temperature and then shifted to incubation at 4°C overnight. The bacteria were then blocked with 3% (w/v) BSA in TBS buffer at room temperature for 1 hour. To access the binding of the proteins to the bacteria, 20 µg of each *Pl*Dscam isoform (with GST fusion tag) or GST diluted in 1% BSA in TBS were added to the wells and incubated at room temperature for 2 h. Following three careful washes with TBS, the bound *Pl*Dscam protein was detected with the GST antibody (1∶2,000) followed by rabbit antimouse HRP-conjugated secondary antibody (1∶3000). After adding 100 µl tetramethylbenzidine or TMB substrate (Sigma) for 20 min and 100 µl of stop solution (0.5 M sulfuric acid), the absorbance of the resulting color was measured at 450 nm. All binding assays were performed in triplicates and experiment was repeated three times.

### Bacteria clearance assay

*E. coli* and *S. aureus* were washed six times in 0.9% NaCl at 1,200× g for 10 min and then incubated with 10 µg recombinant proteins of each *Pl*Dscam isoforms for 1 h at 4°C, followed by washing six times with 0.9% NaCl. One hundred microliter of *E. coli* or *S. aureus* at concentrations of 6×10^8^ and 3×10^9^ CFU/ml, respectively, in CFS were injected into crayfish. The bacteria count was carried out in hemolymph collected 40 min and 3 h after the bacterial injection. The homonym was serial diluted serially and was then dotted onto LB agar (10 µl for each dot) and then incubated at 37°C overnight followed by counting the bacterial colony forming units (CFU).

RETRACTED

### Phagocytosis assay

Both, heat killed *E. coli* and *S. aureus* were conjugated with fluoresce in isothiocyanate (FITC) using a method previously described by Hed [26]. Briefly, heat-killed *E. coli* and *S. aureus* were washed six times in 0.9% NaCl at 1,200× g for 10 min and then incubated at concentration of 10^9^ particles/ml in 0.1 M Na_2_CO_3_ containing 0.1 mg/ml FITC (Sigma), pH 9.5 for 30 min at 37°C, followed by washing six times with 0.9% NaCl as above. The FITC-conjugated heat-killed bacteria were incubated with 10 µg recombinant proteins of each *Pl*Dscam isoforms for 1 h at 4°C. The bacteria were washed five times as described above and resuspended at a concentration of 10^8^ particles/ml in CFS. Two hundred microliter of FITC-conjugated heat-killed bacteria coated with recombinant *Pl*Dscam isoform (4×10^6^ particles/ml in CFS) was injected into the animals via the base of the fourth walking leg. Hemocytes were bled for phagocytosis detection at 1.5 h post FITC-conjugated heat-killed bacteria injection. The fluorescence of FITC-conjugated heat-killed bacteria particles was quenched by adding 20 µl of 0.04% trypan blue (Pfaltz & Bauer, Waterbury, CT). The ingested bacteria were easily detected under the UV light microscope due to their fluorescence. The percentage of phagocytosing cells was determined by counting 10 individual fields and dividing the number of cells with ingested fluorescent bacteria with the total number of counted cells. Each experiment was performed in triplicates.

### Crayfish Hpt cell culture and maintenance

The hematopoietic tissue was dissected according to Söderhäll et al.[27]. The Hpt was washed with CPBS (crayfish phosphate buffered saline: 10 mM Na_2_HPO_4_, 10 mM KH_2_PO_4_, 150 mM NaCl, 10 µM CaCl_2_, and 10 µM MnCl_2_, pH 6.8) and incubated in 600 µl of 0.1% collagenase (type I and IV) (Sigma) in CPBS at room temperature for 45 min to separate the Hpt cells. The separated cells were washed twice with CPBS by spinning down at 800× g for 5 min at room temperature. The cell pellet was re-suspended in modified L-15 medium and subsequently cells were seeded at a density of 2.5×10^6^ cells/150 µl in 96-well plates. The Hpt cells were supplemented with partially purified plasma as a source of astakine [28] after 1 h of attachment at room temperature and the culture plates were incubated at 16°C, and 1/3 of the medium was changed at 48 h intervals.

### Generation of dsRNA

dsRNA of *Pl*Dscam was designed from the conserved region during Ig8-FNIII3. Gene specific primers for *Pl*Dscam and GFP was incorporated with a T7 promoter sequence (italic letters) at 5′ ends (DscamRNAi-F, 5′- *TAATACGACTCACTATAGGG*GCATCAAGCTGAGTGGACAA-3′; DscamRNAi-R, 5′- *TAATACGACTCACTATAGGG* GAAGCCAGGTAGGGGAAATC -3′ and GFP 63+, *TAATACGACTCACTATAGGG* CGACGTAAACGGCCACAAGT; GFP 719-, *TAATACGACTCACTATAGGG* TTCTTGTACAGCTCGTCCATG) and used to amplify PCR products as template for dsRNA synthesis. A GFP transcript was amplified with the pd2EGFP-1 vector (Clontech) as template and used as control. The amplified products were then purified using GenElute Gel extraction kit (Sigma) followed by *in vitro* transcription using the MegaScript kit (Ambion). The dsRNA was purified with the Trizol LS reagent (Invitrogen).

RETRACTED

### RNAi *in vitro* study

The Hpt cells were divided into three groups with four replicates in each group. The Hpt cells received different treatments as follows: group 1: GFP dsRNA plus UV-killed WSSV, group 2: GFP dsRNA plus WSSV and group 3: *Pl*Dscam dsRNA plus WSSV. The dsRNA transfection and WSSV infection into Hpt cell cultures were performed as described by Liu et al.[29]. Briefly, 4 µl of dsRNA (250 ng/µl) was mixed with 3 µl of histone H2A (1 mg/ml) and with 20 µl of modified L15 and added to one well of 1-day-old Hpt cell cultures. The cells were then incubated at 16°C. At day 3, one replicate of group 2 and 3 were subjected to RNA extraction to determine RNAi efficiencies. For remaining replicates, the medium was replaced with 150 µl of L15 medium together with 5 µl of WSSV stock suspension and 5 µl crude astakine preparation and were further incubated for 36 h at 20°C followed by isolation of RNA. Total HPT RNA was extracted to determine *Pl*Dscam and WSSV VP28 transcripts by semi-quantitative RT-PCR. PCR was performed with three oligonucleotide primers (WSSV VP28 (Genbank accession no. AF502435):-F: 5′-TCACTCTTTCGGTCGTGTCG-3′ and -R: 5′- CCACACACAAAGGTGCCAAC-3′; previous primer for 40s ribosomal and *Pl*Dscam gene). The PCR conditions were as follows: 94°C 2 min, followed by 30 cycles of 94°C 20 s, 60°C 20 s, and 72°C 30 s for *Pl*Dscam and VP28, while 25 cycles for 40S ribosomal gene.

### Statistic analysis

The relative expression levels of different time groups were examined by One-way ANOVA followed by Duncan's new multiple range test and Tukey test. Differences were considered statistically significant at *P<0.05*. Results are expressed as the mean ± SE.

## Supporting Information

Figure S1 Variable regions in the cytoplasmic tail of *Pl*Dscam. A) Multiple alignment of amino acid sequence of seven different cytoplasmic tails of *Pl*Dscam. B) Amino acid sequence alignment of the cytoplasmic tail of *Pacifastacus leniusculus* (*Pl*Dscam), *Drosophila melanogaster* (*Dm*Dscam: AAF71926), *Apis mellifera* (*Am*Dscam: AAT96374), *Aedes aegypti* (*Aa*Dscam: EAT37388), *Tribolium castaneum* (*Tc*Dscam: NP_001107841), *Daphnia pulex* (*Dp*Dscam: ACC65888). The squares highlight homologous regions and some conserved motifs are indicated by different colors, including SH3-binding motif (violet), endocytosis motif (yellow), SH2-binding motif (green), Polyproline motif (blue), PDZ motif (red) and ITIM motif (in a box).
(TIF)

Figure S2 Diagram showing the binding locations of primers that were used in this study. The locations of primers that were used for RACE-PCR (A), identification of alternatively expressed regions in *PlDscam* (B) and quantification of PlDscam expression (C).
(TIF)

Figure S3 Dscam is important for phagocytosis of crayfish hemocytes. Phagocytosis of FITC-conjugated heat killed *E. coli* or *S. aureus* particles were determined using normal or UV light microscopy. A) phagocytosis of FITC conjugated heat-killed *E. coli* after pre-incubation with different isoforms (N2, E6 or S9) of recombinant proteins of *Pl*Dscam. B) phagocytosis of FITC conjugated heat-killed *S. aureus* after pre-incubation with different isoforms (N2, E6 or S9) of recombinant proteins of *Pl*Dscam. The white, black and red arrows represent ingested FITC-conjugated heat-killed bacterial particles, nodule formation and nodules that contain several ingested bacterial particles, respectively.
(TIF)

Table S1 Primer pairs used in this study. All primer sequences are given in the format 5′-sequence-3′.
(DOC)

Table S2 Comparison of Dscam Ig2 and Ig3 combinations in normal, *E. coli* injected and *S. aureus* injected crayfish. Fifty individual cDNAs, expressed in each group, were sent to sequence.
(DOC)

Table S3 The chosen clones were used for construction of the clustering phylogram and the clones in bold letters were expressed as recombinant proteins.
(DOC)
